The article "N-GPETS: Neural Attention Graph-Based Pretrained Statistical Model for Extractive Text Summarization" was retracted in 2023. Reasons: signs of a paper mill; compromised peer review; unreliable results or conclusions.

# N-GPETS: Neural Attention Graph-Based Pretrained Statistical Model for Extractive Text Summarization

**DOI:** 10.1155/2022/6241373

**Published:** 2022-11-22

**Authors:** Muhammad Umair, Iftikhar Alam, Atif Khan, Inayat Khan, Niamat Ullah, Mohammad Yusuf Momand

**Affiliations:** ^1^Department of Computer Science, City University of Science and Information Technology, Peshawar 25000, Pakistan; ^2^Department of Computer Science, Islamia College, Peshawar 25000, Pakistan; ^3^Department of Computer Science, University of Engineering and Technology, Mardan, Pakistan; ^4^Department of Computer Science, University of Buner, Buner 19290, Pakistan; ^5^Faculty of Computer Science, University of Nangarhar, Jalalabad 2600, Afghanistan

## Abstract

The extractive summarization approach involves selecting the source document's salient sentences to build a summary. One of the most important aspects of extractive summarization is learning and modelling cross-sentence associations. Inspired by the popularity of Transformer-based Bidirectional Encoder Representations (BERT) pretrained linguistic model and graph attention network (GAT) having a sophisticated network that captures intersentence associations, this research work proposes a novel neural model N-GPETS by combining heterogeneous graph attention network with BERT model along with statistical approach using TF-IDF values for extractive summarization task. Apart from sentence nodes, N-GPETS also works with different semantic word nodes of varying granularity levels that serve as a link between sentences, improving intersentence interaction. Furthermore, proposed N-GPETS becomes more improved and feature-rich by integrating graph layer with BERT encoder at graph initialization step rather than employing other neural network encoders such as CNN or LSTM. To the best of our knowledge, this work is the first attempt to combine the BERT encoder and TF-IDF values of the entire document with a heterogeneous attention graph structure for the extractive summarization task. The empirical outcomes on benchmark news data sets CNN/DM show that the proposed model N-GPETS gets favorable results in comparison with other heterogeneous graph structures employing the BERT model and graph structures without the BERT model.

## 1. Introduction

The rise of the Internet and big data results in a massive and exponential growth of information. Because of this, numerous academics are working to develop a technical method for automatically summarizing texts. The automatic summarization approaches generate summaries containing the relevant information from the input documents to review it quickly without compromising its originality [1]. Extractive and abstractive are the two types of summarization. A subset of sentences from the input text is chosen through extractive summarization to provide a summary [2]. In contrast, abstractive summarization restructures the language in the text and, if necessary, introduces new words/phrases into the summary. In general, extractive summarization models are simple, and they express the summarization task as a classification problem for document sentences: whether or not to include it in a summary [3].

The neural sequence-to-sequence encoder-decoder framework has demonstrated incredible performance doing extractive summarization in the past few years. In research [4], researchers design an encoder that works hierarchically and summarize single-document text. They employ an extractor, which works on an attention mechanism allowing to extract sentences or words from documents for summarization tasks. The study [5] proposed a neural extractive summarization model as a sentence ranking task, incorporating a reinforcement learning objective to optimize the ROUGE evaluation metric. Encoder-decoder sequence architecture for extractive summarization was mostly adopted by the researchers [6–8] who utilize various neural components to encode each sentence uniquely. To produce a summary from the input content that includes significant sentences, learning and modelling cross-sentence linkage are crucial [9]. Recurrent neural networks (RNNs) have been used in the majority of the recently presented research, including [4, 10, 11], to learn and simulate the cross-relationships between texts. However, RNNs may suffer from the vanishing gradient problem, which causes gradient magnitudes to shrink as they propagate over time. Because of this phenomenon, the network's memory ignores long-term dependencies and fails to learn the correlation between temporally distant events [12].

To understand and simulate the cross-relationship between sentences, many scholars took advantage of the graph structure. There have been numerous attempts made to model effective graph networks for jobs requiring summarization [9]. Recent research [12] used sentence personalization traits and discourse-aware intersentential interactions to create a summarization model (ADG). The authors in [13] used a Rhetorical Structure Theory (RST) graph to model cross-sentence association by utilizing joint extraction and syntactic compression to create a summary of a single-document text. Another approach is proposed in [14], where a different strategy is suggested. It looks at an unsupervised discourse-aware hierarchical graph network (HIPORANK) for lengthy scientific publications, which uses intra- and interconnection between document sentences as well as model asymmetric edge weights for extracting important sentences.

The preceding approaches relied on third-party tools and did not consider the error propagation problem [9]. One of the simplest methods mentioned above is to model a fully connected graph at the sentence level. Recently, studies [6, 7] used transformer architecture to learn pairwise interactions between phrases to model sentence-level graphs. A hybrid graph attention framework for learning the cross-sentence relationships was put forward by [8] utilizing GAT and CNN as encoders while TF-IDF values as edge features. However, this graph-building approach runs into the problem of capturing semantic-level relationships [14]. In a study [14], the authors developed a sentence-level graph-based model that employed BERT for sentence encoding and a joint neural network model (NTM) to discover latent topic information rather than semantic word nodes in a heterogeneous graph network. The authors in [15] proposed a heterogeneous graph structure for modelling the cross-sentence relationships between sentences. They used three types of nodes to capture the relationships between the EDUs: nodes of the sentence, nodes of EDU, and nodes of entity, RST, and they also used external discourse knowledge to improve the model's results. The creation of a useful graph model that enhances the extraction of important stuff for the formation of extractive summaries remains a challenging and unsolved research issue despite the success of the prior approaches [9].

This paper suggests an innovative pretrained statistical-based graph attention network (N-GPETS) for single-document extractive summarization, fusing BERT pretrained framework and TF-IDF with graph attention network. First, the whole document is fed to BERT for encoding, which has a strong architectural foundation and has been pretrained on enormous data sets. The BERT encoder generates word nodes and sentence nodes. These word nodes served as an additional semantic unit. Second, for the graph layer, the output of the BERT encoder in the form of word and sentence nodes act as graph nodes while the values of TF-IDF of the whole document serve as edge features between corresponding nodes. In graph layer, the graph attention mechanism is applied and the representation of nodes ware updated. Finally, labels are assigned by the sentence selection module after it has extracted the representation of significant sentences node from the graph layer.

N-GPETS enhanced the work of [9], which was actually about the problem of capturing semantic-level relationships, but this work was completely unaware of using pretrained models such as BERT along with graph attention mechanism. N-GPETS also differs from previous work [14] as they use topic nodes as an additional semantic unit with the help of a joint neural network model (NTM). The other difference of proposed N-GPETS from previous models is to generate TF-IDF values of the whole input text and used these features between edges of graph nodes. The proposed N-GPETS graph structure has the following advantages: (i) during the graph propagation stage, semantic word nodes (additional units) which are highly featured rich, due to the BERT framework [16], improve the sentence representation and gather information from sentences; (ii) to link sentences and identify intersentence links, semantic word nodes can also be employed as a bridge; and (iii) our graph structure can use different levels of information during message passing. The following are our model's standout contributions:

1. a novel approach and first attempt to build a BERT-based statistical graph attention network N-GPETS for summarizing single-input document text. An extractive summary is produced by the graph layer using sentence and word nodes produced by BERT and TF-IDF values of the entire manuscript.
2. to assess the effectiveness of the suggested N-GPETS technique against cutting-edge approaches using CNN/DM News data sets using ROUGE evaluation metrics.
3. The simulation findings on benchmark news data sets: CNN/DM demonstrates that N-GPETS provides generally acceptable outcomes in comparison with existing graph attention networks utilizing BERT or the absence of BERT in combination with graph structures.

The remaining portions of the article are organized as follows. In Section 2, we take a critical look at the leading work on extractive summarization tasks.  Section 3 describes in full the proposed N-GPETS model methodology.  Section 4 details the proposed model compared to other existing cutting-edge models and also the hyper-parameters and model settings.  Section 5 focuses on Results, and lastly, the study paper concludes in section 6, which also offers suggestions for future research.

## 2. Literature Review

This section discusses some traditional and advanced approaches/techniques for extractive summarization tasks. Initially, we look into how extractive summarization is performed using a deep neural sequence-to-sequence model. Then, we investigate how various statistical methods, such as TF-IDF, LDA, and TextRank, perform feature extraction and summary generation tasks. Then, deep-learning-based transformer architectures for extractive summarization are presented. We discuss how pretrained models, such as BERT, are used for various NLP tasks, particularly summarization. Finally, we look into how other neural graph-based structures are used for the task of summary generation. In the following section, we will briefly define some background concepts.

### 2.1. Text Summarization

Automatic text summarization (ATS) is a method that creates an overview that contains all pertinent and important information by automatically summarizing a substantial amount of text. It is important to note that automatic text summarization is a text mining process that accepts a lengthy text document as input and produces an appropriate summary [17]. There is an abundance of text-based content on the Internet, including web publications, papers, news, and reviews, that must be summarised to get the document's gist [18]. ATS has many uses, such as short read generation, passage reduction, compaction, extracting, and the most important information from sensitive reports, including legal reports produced by legal authorities [19]. ATS can also be used in news text summarizers to assist readers in finding the most interesting and important content in less time [20–22]. Other applications of ATS include sentiment summarization, legal text summarization, scientific document summarization, tweet summarization, book summarization, story/novel summarization, e-mail summarization, and bio-medical document summarization [23]. The fundamental design of the ATS system, as shown in Figure 1, includes the following functions.

- The Transformer is a fully self-attention-based deep learning model. It is a simple network that is completely free of recurrence and convolutions. It is one of the most advanced architectures in NLP and computer vision [12]. The Transformer does not need to comprehend the initial part of the sentence before the end because the attention mechanism adds context to the input sequence at any point in the sentence. Instead of processing input sequentially as RNN does, the Transformer allows for more parallelization, which results in a shorter training time. Because of Transformer's parallelization feature, training on larger data sets is possible, allowing for the development of cutting-edge pretrained models such as BERT (Bidirectional Encoder Representations from Transformers) and GPT (Generative Pretrained Transformer) trained on massive corpora [12, 24].
- BERT (Bidirectional Encoder Representations from Transformers) is a Google-developed machine learning model that has already been trained for natural language processing (NLP) tasks. The Google AI research team created and published BERT in 2018. It should be noted that Google announced in 2019 that their search engines are using the BERT approach. In 2020, one of the most recent surveys [24] claims that BERT in just one year has evolved into a widely used baseline in NLP research, with over 150 research publications analyzing and improving the model. BERT is a new language representation baseline that extends word embedding models [25]. Two significant duties were covered in BERT training: language modelling (15% of tokens were hidden, and BERT was taught to anticipate them based on context) and next sentence prediction (using the first sentence as a guide, BERT was trained to determine whether a particular statement would be expected or not).
- *Graph Attention Networks* (GATs). To address the limitations of earlier methods that just used graph convolutions, neural network designs called graph attention networks (GATs) deal with input that is arranged as a graph and employ masked self-attention layers [26]. By focusing on each node's neighbors, it is intended to employ a self-attention method to calculate each node's hidden representations. Some of the most useful characteristics of the graph attention architecture include the following: (i) the parallelization characteristic is surrounded by node-neighbor pairs, which makes the attention mechanism effective. (ii) By giving the neighbors different weights, this architecture is especially efficient because it can be used with graph nodes of different degrees. (iii) The graph attention model can be used to directly address learning issues, such as those requiring the model to extrapolate to previously unobserved graphs [26].

### 2.2. Extractive Text Summarization Approaches and Techniques

Finding the sentence's location and the frequency of words in the text was the most typical problem that surfaced from extractive summarization research [1]. Researchers in [27] used a deep learning technique called Feed Forward Neural Network (FFNN) for single-document legal text summarization. This method generates a coherent extractive summary without needing features or domain expertise but fails miserably in summarizing difficult and long statements [1]. The study [11] presented the encoder-decoder architecture as a foundation for single-document summarization that contains an attention-based extractor and a hierarchical document encoder. The authors in [28] presented a classifier-based architecture (RNN based) that accepts or rejects each sentence in the original document order for inclusion in the final summary in a sequential manner. For a lengthy text that takes into account both the global and local contexts of the content, the authors of [29] suggested a single-document extractive summary model. A novel technique for summarization was provided by the authors in [30] that relied on a neural sequence-to-sequence model with an attention mechanism and fuzzy characteristics that could be customised.

Statistical techniques such as TF-IDF, TextRank, LDA, and clustering, among others, have been used for extractive summarization tasks. The study [31] presented statistical topic modelling techniques such as latent Dirichlet allocation (LDA), which select important sentences in clusters based on automatically generated keywords. Additionally, the study in [32] mainly utilized TF-IDF and K-means clustering-based approaches for the creation of an extracted summary.

The authors in [33] presented two methods for extractive summarization of hotel reviews. The first method was used to select the most related sentences based on their TF-IDF score. The second method generated the phrase summary style by pairing adjectives with the closest nouns and taking polarity into account. The work done by [34] integrated the TF-IDF and TextRank techniques to extract keywords from input documents.

A deep learning model called Transformer uses the self-attention process. This framework is utilized by numerous researchers for extractive summarization jobs. The researchers of [35] focused on the structured transformers HiBERT presented by [36] and Extended Transformers presented by [37], which offer an extractive encoder-centric stepwise strategy for summarizing documents. This model enabled stepwise summarization by inserting the previously created summary as an additional substructure into the structured Transformer. The authors in [38] presented an extractive summarization model based on layered trees, where the given document's discourse and syntactic trees are combined to form nested tree structures. The authors primarily focused on the existing model RoBERTa presented by [39] for constructing this model. By lowering the size of the attention module, the authors in [40] presented an extractive summarization technique for discourse-based attention at the document level; this constitutes the core of the transformer architecture, utilizing a unique discourse-inspired approach. Two different transformer-based techniques for sentiment analysis were provided by the authors in [41] while fetching the words that are crucial to the model's decision-making to produce a summary as the output explanation. To generate unsupervised extractive summaries, the researchers of [42] used a transformer attention mechanism to prioritize sentences. For extractive summarization of long text, the authors of [43] used the transformer model and introduced a type of heterogeneous framework called HETFORMER framework. BERT is a pretrained model used by many researchers for extractive summarization. The summarized literature review is depicted in Table 1.

The “lecture summarizing service,” a Python-based RESTful service, chose relevant sentences near the cluster's centroid using the K-means clustering algorithm and the BERT model for text embeddings to generate a summary [47, 48]. Researchers in [49] utilize the bidirectional model BiLSTM and BERT model for extracting temporal information from messages from social media platforms that are necessary for geographical applications. The authors of [50] developed a hybrid method for producing summaries of long scientific texts that combined the benefits of both extractive and abstractive designs. The authors in [51, 52] use the deep learning model BERT and RISTECB model to answer important questions related to the COVID-19 research articles. The authors of [44] demonstrated an excellent tuning-based approach for extractive summarization using the BERT model. The BERT model was also used by the authors of [7, 8, 16, 36, 46] for contextual representation in summarization tasks. The authors in [53] use the BERT model to automatically generate titles from a huge set of published literature or related work. Additionally, extractive summarization tasks using graph structures have been carried out by exploiting linguistic and statistical information included in sentences [9]. Recent research has combined neural networks with graphs, or (GNNs), and used the encoder-decoder structure for extractive summarization [13, 54]. Many researchers nowadays use a heterogeneous graph neural network with multiple updated nodes rather than a homogeneous graph structure with no updated nodes for extractive summarization tasks. The study [55] proposed a bipartite graph attention network for multihop reading comprehension (RC) across documents that encoded different documents and entities together. The authors in [48] presented an approach that modeled redundancy-aware heterogeneous graphs and refined sentence representation using neural networks for extractive summarization. The studies [9, 56] proposed a heterogeneous graph neural network for extractive summarization that used CNN with Bi-LSTM as encoders for input text and TF-IDF values as edge features between graph nodes. Utilizing a graph attention network, cross-sentence links between sentences are learned. The work done by [14] built a sentence-level graph-based model, using BERT for sentence encoding and joint neural network model (NTM) for discovering latent topic information. The authors in [15] proposed a heterogeneous graph structure for modelling cross-sentence relationship between sentences. To represent the relationships between the EDUs, they used three different types of nodes, including sentence nodes, EDU nodes, and entity nodes, and RST discourse parsing and leverage external discourse expertise to enhance the model's performance. The next section goes over the unique model N-GPETS methodology that is proposed in this study in depth.

## 3. Methodology

In this paper, an innovative pretrained statistical model for extractive summarization task called N-GPETS is presented, which is designed by combining the deep learning model BERT and graph attention network along with a statistical approach. N-GPETS is broken down into four phases: document representation comes first, then there are three trainable modules: BERT graph initializers, graph layer, and important sentences selector. The following subsections go over each of these phases in detail.

### 3.1. Representing Document as a Heterogeneous Graph

Consider a document represented by *G* = (*V*, *E*), where *V* represents the set of nodes, and *E* represents the edges in between the nodes. In our framework, the attention graph structure is made by taking the union of *V*_*W*_ and *V*_*S*_, i.e., *V*=*V*_*W*_*UV*_*S*_, *E*=*e*_11_,…, *e*_*mn*_, and *V*_*W*_=*W*_1_, *W*_2_,…, *W*_*m*_. The quantity of distinct words in the text *V*_*S*_=*S*_1_, *S*_2_,…, *S*_*n*_ indicates the quantity of sentences. *E* is now an edge weight matrix with real values and *e*_*ij*_ ≠ 0 where *i* ∈ {1,…, *n*} and *j* ∈ {1,…, *m*} demonstrate that *j*_th_ sentence has the *i*_th_ word as discussed in [9].

According to Figure 2, three primary trainable modules make up the N-GPETS: BERT graph initializers, graph layer, and important sentences selector. The N-GPETS model works as follows: first, the pretrained BERT graph initializer module generates sentence and word nodes using the BERT encoder as opposed to alternative neural network encoders already employed in other works. These word and sentence nodes are then transmitted to the graph layer for the document graph together with the TF-IDF values utilized as edge characteristics. The heterogeneous graph layer uses the graph attention network to relay messages between these word and sentence nodes in the second step, iteratively changing these nodes as a consequence. Finally, the important sentence selection module extracts the final summary's important sentence nodes.

### 3.2. BERT Graph Initializers

As suggested by the BERT model's basic structure, the output vectors of BERT are based on tokens instead of sentence tokens [25]. But it is clear to us that sentence-level representation is manipulated in the case of extractive summarization. The second thing that was noted was that the original BERT model's segmentation embeddings just apply to the input of two sentences. Nevertheless, the extractive summarization process requires us to encode and manage multisentential inputs [7]. In this study, each sentence begins with a [CLS] external token and ends with a [SEP] that overcomes the difficulties that arise for single sentence representation in a document, same as done in [7]. For the preceding sentence, external tokens gather data while to differentiate different sentences in a document, segment embeddings are used [7]. For example, we have five different sentences in an input text, i.e., (sent_1_, sent_2_, sent_3_, sent_4_, and sent_5_). Each sentence has the following embeddings associated with it: [EA, EB, EA, EB, and EA]. This method allows for the hierarchical learning of the input document representations. In last, the vectors *T*_*i*_ which are the vectors of [CLS] tokens of every sentence generated by BERT having all information about each sentence sent_*i*_ are forwarded to the graph layer for the graph attention mechanism. These vectors work as sentence nodes in the graph layer in the proposed N-GPETS. The complete process of sentence nodes generation using BERT is depicted in Figure 3 [44].

### 3.3. Word Nodes and Edge Features

We employ the base framework of the BERT encoder [25], depicted in Figure 2, which takes the word of input text, encodes the words, and generates word vectors. To highlight how word and sentence nodes are connected, in the initialization step of our model, we incorporate TF-IDF values into the edge weights, similar to [9]. Utilizing BERT to create word, nodes are presented in Figure 4.

### 3.4. Overview of the BERT Graph Initializers Phase

- Nodes of sentences creation (*T*_*i*_)
- Nodes of words creation
- These sentence vectors, word embeddings, and TF values of the whole input text are forwarded to the attention graph layer
- The graph layer serves as a summarization layer in the N-GPETS model

### 3.5. Graph Layer

In the graph layer for the construction of a bipartite graph, we gave the nodes of words and sentences along with TF values to the graph layer. After that to update the representation of the semantic nodes, the graph attention network is used, same as previous work [9], with the main difference being that the word and sentence node features used in the graph layer are encoded with the help of BERT model at the graph initializers stage discussed above rather than using different neural network encoders such as CNN or Bi-LSTM. The graph attention layer (GAT) and hidden state of input nodes *h*_*i*_ ∈ *R*^dh^ can be constructed in the same way as demonstrated in [9]:

(1) zij=LeakyReLUwawqhi;wkhj,αij=expzij∑l∈Niexpzil,ui=σ∑j∈NiαijWvhj.

Here, *w*_*a*_, *w*_*q*_, *w*_*k*_, and *w*_*v*_ denote training weights and attention weight across *h*_*i*_ and *h*_*j*_ denoted by *α*_*ij*_. Following is the illustration of multihead attention [9]:

(2) $$\begin{array}{c} u_{i}=\left\|\right)\underset{k=1}{K}\sigma \left(\sum_{j\in N_{i}}\alpha_{ij}^{k}W^{k}h_{i}\right). \end{array}$$

The resultant output representation is as follows [9]:

(3) $$\begin{array}{c} h_{i}^{\prime }=u_{i}+h_{i}. \end{array}$$

Now, equation (1) is changed to include edge weights *e*_*ij*_ in graph attention layer, which is given as follows [9]:

(4) zij=LeakyReLUWaWqhi;Wkhj;eij.

### 3.6. Iteratively Updated Nodes

The information propagation is used to send messages between the nodes of words and sentences. Specifically, after initialization, we use the GAT and FFN layers to change sentence nodes with their neighbor nodes of words. Then, using updated sentence nodes, we obtain new representations for word nodes and iteratively update sentence nodes. Each iteration includes both a sentence-to-word and a word-to-sentence update process. The process can be represented for the *t*th iteration [9].

(5) $$\begin{array}{c} U_{s\leftarrow w}^{t+1}=\text{GAT}\left(H_{s}^{t},H_{w}^{t+1},H_{w}^{t+1}\right),\\ H_{s}^{t+1}=\text{FFN}\left(U_{s\leftarrow w}^{t+1}+H_{s}^{t}\right). \end{array}$$

### 3.7. Sentences Selection Module

Finally, the sentences selection module selected those important sentence nodes from the graph layer which become the part of the final extractive summary produced by the proposed model. For this task, node classification is done, which predicts labels 0 or 1 for each sentence in a document and cross-entropy loss as the overall system's training objective. Those sentences having label 1 include in the final summary while sentences with label 0 are not included in the final summary.

## 4. Performance Evaluation

This segment evaluates the performance of the suggested N-GPETS architecture to other latest models for the extractive summarization job. This section covers the dataset utilized in the proposed work and compares BERT-based and non-BERT models to the suggested model and also provides information about the objective evaluation matrices utilized in the proposed system, as well as its hyperparameters and execution settings. The following subsections described them in a little bit of detail:

### 4.1. Objective Evaluation Matrices

The matrices like precision, recall, F-measure accuracy, and ROUGE toolkit are adopted by state of the art [9, 57–59]. They are defined below.

#### 4.1.1. Precision

The number of sentences appearing in both the system and the abbreviations for reference divided by the number of sentences present in the summary produced is called precision (*P*) [57].

#### 4.1.2. Recall

Recall (*R*) is the number of sentences from both produced systems and reference abbreviations divided by the number of sentences present in the reference summary [57].

#### 4.1.3. *F*-Score

The *F*-score is a compact matrix that combines accuracy with memory. Calculating the corresponding measure of accuracy and memory is a basic method for calculating the effect of the *F*-score [57, 58].

#### 4.1.4. Accuracy

Accuracy is the total number of well-labeled sentences divided by the number of sentences present in the data set test set.

#### 4.1.5. N-Gram Co-Occurrence Statistics—ROUGE

ROUGE stands for Recall-Oriented Understudy for Gisting Evaluation proposed by [58] is the most commonly used testing tool in text summary research. This system compares the quality of the summary produced by the system with the man-made summary to determine how good it is. The gold standard we used includes two personal abbreviations and two human quotes. ROUGE test steps include ROUGE-N (*N* = 1, 2, 3, and 4) and ROUGE-L, ROUGE-W, ROUGE-S, and others. ROUGE-N quantifies the number of 'n-gram' matches between system summary and set of human summaries.

### 4.2. Data Set

This study examined N-GPETS using a CNN/Daily Mail (anonymous version) data set, a standard data for marking news [60]. The data set is classified and processed according to standard classification, with 287,227/13,368/11,490 examples (92.5%/4.2%/3.6%) for training, validation, and sequence of tests, respectively, similar to previous tasks [7, 9, 14, 15]. CNN/Daily Mail data set statistics are set out in Table 2 [14].

### 4.3. Models for Comparison

The N-GPETS model compares high-resolution BERT-based graphs with non-BERT neural graph models for extracting text.  Table 3 presents the details of the non-BERT graph structures, and Table 4 shows the graph properties using the BERT model.

#### 4.3.1. Hyperparameters and Implementation Settings

N-GPETS encodes the document using a pretrained BERT-based model to produce sentence and word nodes. Vocabulary is limited to 50,000 words, and tokens are activated in 300-dimensional embedding using BERT than the embedded GloVe used in previous applications [7, 9]. The BERT output is 768-dimensional vectors, and the tokens are 256-dimensional vectors.

Since the output of BERT is 768-dimensional vectors and the tokens taken by the Graph layer should be equal to the 300-dimensional embedding as described in [8], we use a linear layer after the BERT output that converts the 768-dimensional vector to a 300-dimensional vector. When you create word nodes, stops and punctuation are filtered. We limit the length of a sentence to 50 characters. To address the problem of common noisy words, we remove 10% of vocabulary from databases with low TF-IDF values. To start a sentence node, the maximum size is kept at d*s* = 128, and the maximum size of the *e*_*ij*_ edge elements is kept at d*e* = 50. FFN is 512. Deep Graph Library (DGL) is used to use the graph neural network, as is the case with [9].

Thirty-two batch size is used in training, and Adam's provided [50] with a reading rate of 5 and 4 is used. Premature stops are made when the allowable loss is not less than three consecutive epochs. Based on the functionality of the verification set, the number of duplicates is set to *t* = 1. N-GPETS selects the top three sentences as a system-based summary of the average length produced by human beings on CNN/Daily Mail, three sentences. The specification of the system in which we train our model is 8 GB Random-Access Memory (RAM) and Intel (R) Core (TM) 7-6600U. The CPU is based on ×64 architecture and uses a 64-bit operating system. The Windows operating system installed is Windows 10 Pro.

## 5. Results and Discussion

This section outlines the overall empirical findings generated by our suggested model, N-GPETS. N-GPETS is evaluated using the criteria that when compared to other models, does N-GPETS, which generates sentence and word nodes using BERT encoder and also has TF-IDF connections between nodes, produce adequate results? First, a frequently used CNN/DM data set is utilized to train and then test the N-GPETS model. For reference summaries, we considered the unigram R-1, bigram R-2, and longest common subsequence R-L overlap. Second, a comparison has been made between the proposed framework N-GPETS and previously working both BERT-based and non-BERT graph structures as depicted in Section 4.3. Additionally, ablation research is carried out to show the importance of each model element.

### 5.1. Overall Performance

On the CNN/DM data set, Table 5 displays the ROUGE *F*-scores for several models. This table is divided into four sections: the first section contains the Lead-3 and Oracle scores, the second section contains the scores of models that did not use BERT, the results of BERT-based models are contained in the third part, and the findings of the suggested model N-GPETS are shown in the fourth part. The results lead to the following conclusions: N-GPETS performs better than the cutting-edge non-BERT model HSG by a 1.8/1.3/2.2 on the *F*-score of R-1/R-2/and R-L. This shows that our graph network, which is based on the BERT algorithm, has a better comprehension of learning cross-sentence links. Additionally, N-GPETS performs better than each of the non-BERT models presented in Table 5. After that comparison to models that utilized BEET, first, N-GPETS is contrasted with Topic-Graph-Sum, which utilizes topic data via NTM as an additional semantic unit. N-GPETS produced better results beating the Topic-Graph-Sum framework by 0.13/0.05/0.42 on the *F*-score of R-1/R-2/R-L. Second, when compared to BERTSum-sent, N-GPETS achieves better results having an increase of 0.9/0.62/1.03 on the *F*-score of R-1/R-2/R-L. Third, in contrast to DiscoCorrelation-GraphSum, which captures relationships between EDUs via entity nodes, EDU nodes, and RST discourse parsing, N-GPETS shows better outcomes on ROUGE R-1/R-2 having an increase of (0.54/0.05), respectively, and having the same score on R-L.

It should be mentioned that RST discourse parsing and third-party external tools are the foundation of DiscoCorrelation-GraphSum. Contrarily, N-GPETS does not utilize any outside tools or knowledge. Additionally, N-GPETS beats the cutting-edge extractive summarization model DISCOBERT depended on the external tool in R1 metrics and produces results that are equivalent in R2 and RL metrics.

### 5.2. Ablation on CNN/Daily Mail

To understand the function and impact of various contributed modules revealed in our recommended model N-GPETS on performance, ablation research is conducted. First of all, the residual connections that are present between GAT layers were removed and word nodes were attached to the initial sentence feature, similar to previous work [9]. The second thing that we have done, rather than using TF-IDF values from the entire document, TF-IDF values from the individual sentences were used as features in the graph layer. In the third one, we gave a sideline to the BERT model and make use of BiLSTM and CNN models for encoding the document and checking the overall performance. According to Table 6, cutting off residual connections between GAT layers lowers the *F*-score for the R1/R2/and RL measures. This implies that residual connections are crucial in integrating genuine representation with messages updated from other sorts of nodes that cannot be substituted by straightforward concatenation [8]. As shown in Figure 5, we noticed a decline in the *F*-score of R1/R2/RL metrics when TF-IDF values (computed from individual sentences) were used as edge features in the graph layer, demonstrating the effectiveness of TF-IDF values the entire document. Lastly, by substituting CNN-Encoder and BiLSTM in place of the BERT model, the model achieves lower *F*-score values than the proposed model N-GPETS, and the model is reduced to the HSG, a non-BERT model [9].  Figure 6 shows ROUGE-2, *F*1 findings on the CNN/DM data set for our full model N-GPETS, and three ablated variations.

### 5.3. Environment for Model Development and Training

Due to its superior GPU compared to the free version, Google Colab (pro) is utilized for model coding and training instead of using simple COLAB. Programmers can write and execute Python code directly from their browsers using Colab, a Google Research product. It is important to note that Google Colab is a great tool for a variety of deep learning jobs. The Jupyter notebook is hosted by Google Colab. Consequently, no additional software is needed. The advantages of Google Colab include preinstalled libraries and the capacity to upload files to the cloud. With the help of the COLAB collaboration tool, several developers can collaborate on the same project and use free GPUs and TPUs. We train our model for five epochs on 287000 CNN/DM news articles.  Figure 7 shows examples of summaries generated by proposed model N-GPETS along with reference summaries.

## 6. Conclusion and Future Work

The process of creating an extractive summary relies heavily on modelling the relationships across the input sentences. Inspired by the popularity of Transformer-based Bidirectional Encoder Representations (BERT) pretrained linguistic models and graph attention network (GAT) that captures intersentence associations, this study proposes a novel neural model (N-GPETS) for extractive summarization task by combining heterogeneous graph attention network with BERT model and statistical approach using TF-IDF values. In contrast to earlier research, nobody employed BERT for both sentence and word node formation along with the TF values for the creation of an attention graph network. The following benefits are associated with constructing the N-GPETS model: (i) during graph propagation, the addition of feature-rich semantic word nodes encoded using BERT strengthens sentence representation. It can compile information from modified sentences. (ii) Additionally, semantic word nodes can be used to link sentences together and identify links between them. (iii) Our graph structure can use different levels of information during message passing. According to the simulation findings on the widely used CNN/Daily Mail benchmark data set, our model performed better than other heterogeneous graph structures that used the BERT model as well as graph structures that are opposed to BERT. N-GPETS is based on the summarization of a single document. However, it can be expanded to include summarizing numerous documents rather than just one. Using this graph structure to condense lengthy research publications is the second direction for the future. Other semantic units like topic and paragraph semantic units in graph structure can also be used to improve summarization performance.

## Figures and Tables

**Figure 1:** ATS basic architecture for single and multidocument [23].

**Figure 2:** A general framework of the suggested model (N-GPETS).

**Figure 3:** Using the BERT model for extractive summarizing [44].

**Figure 4:** Utilizing BERT to create word nodes [25].

**Figure 5:** ROUGE-1, *F*1 findings on the CNN/DM data set for our full model N-GPETS, and three ablated variations.

**Figure 6:** ROUGE-2, *F*1 findings on the CNN/DM data set for our full model N-GPETS, and three ablated variations.

**Figure 7:** Examples of summaries generated by proposed model N-GPETS along with reference summaries.

**Table 1:** Literature review.

Author(s)	Research technique(s)	Data set
Huang et al., 2021 [15]	BERT, graph attention network (GAT)	New York Times (NYT) data set. CNN/Daily Mail data set.
G. N. H, R et al., 2021 [33]	TF-IDF, combining adjectives	TripAdvisor website
Approach et al., 2021 [41]	Transformer, attention mechanism	IMDB Large Movie Review data set
Peng Cui et al., 2020 [14]	BERT, joint neural network model (NTM) graph attention network (GAT)	New York Times (NYT) data set.
		CNN/Daily Mail data set.
		PubMed and ArXiv data sets.

Wang et al., 2020 [9]	CNN + BiLSTM encoders, TF-ID, heterogeneous graph attention network	New York Times (NYT) data set
		CNN/Daily Mail data set
		Multi-News data set

Hernandez et al., 2020 [31]	LDA latent Dirichlet allocation, TF-IDF, N-Grams, clustering	DUC 2002 data set
Anand et al., 2019 [27]	Feed-forward neural network.	Indian supreme court judgment document
Zhou et al., 2018 [11]	RNN, encoder-decoder architecture.	CNN/Daily Mail data set
Khan et al., 2019 [32]	TF-IDF, K-means clustering	News headlines data set
Xu et al., 2019 [13]	BERT, RST graph, Coreference graph, graph convolution network	New York Times (NYT) data set
		CNN/Daily Mail data set

Narayan et al., 2020 [35]	Structured transformer model	CNN/Daily Mail data set
Liu et al., 2019 [44]	BERT + LSTM, BERT + Transformer	New York Times (NYT) data set
		CNN/Daily Mail data set

Liu and Lapata et al., 2019 [7]	BERT + Transformer model, encoder-decoder framework	New York Times (NYT) data set
		CNN/Daily Mail data set
		XSum data set

Linmei Hu et al., 2019 [45]	Semi-supervised, heterogeneous graph attention network, dual-level attention mechanism	AGNews data set
		Snippets data set
		Ohsumed data set
		TagMyNews data set
		PTE data set
		TextGCN data set
		HAN data set

Jiacheng Xu et al., 2019 [46]	BiLSTM, convolution neural network (CNN), feed-forward neural network (FFNN)	New York Times (NYT) data set
		CNN/Daily Mail data set

Zhang et al., 2018 [36]	Unsupervised method, BERT + Transformer	New York Times (NYT) data set
		CNN/Daily Mail data set

Nallapati et al., 2016 [28]	RNN classifier-based framework	DUC 2002 data set
		CNN/Daily Mail data set

**Table 2:** CNN/Daily Mail data set statistics.

Data set	Source	#Docs			#Avg. tokens	
		Train	Val	Test	Doc.	Sum.
CNN	News	90,266	1,220	1,093	761	46
Daily Mail	News	196,961	12,148	10,397	653	55

**Table 3:** Non-BERT graph structures.

Author(s)	Model name	Non-BERT graph structure
Zhou et al., 2018, [11]	NeuSum	A framework based on the attention of seq2seq to extract text summary.
Wang et al., 2020, [9]	HSG	A model based on a variety of abstract graphs forms a graph of a sentence document based on word appearance. These words and sentence coding notes are CNN and BiLSTM.
Xu et al., 2020, [13]	JECS	The compression model selects sentences and, to reduce repetition, suppresses these sentences by pruning the dependency tree.
Crawford et al., 2018, [61]	BanditSum	Faces the problem of selecting sentences as a contextual problem. To train model policy, gradient methods are used.

**Table 4:** BERT-based graph structures.

Author(s)	Model name	BERT-based graph structure
Liu et al., 2019, [44]	BERTSum (sent)	It uses several separating tokens in documents and gets sequential sentence representations. It should be noted that this model was the first BERT-based model for extraction operations. We and many other functions use its framework as a document encoder.
Zhang et al., 2018, [36]	HiBERT	First, it works by transforming the BERT structure into a sequential structure and then using the unattended to train it in advance.
Xu et al., 2019, [46]	DISCOBERT	One of the most modern abstraction models uses the BERT model to assemble sentences and update these sentence presentations with the help of a graph. It is clear that DISCOBERT only uses sentence beginning and endings. However, we use sentence verbs and additional semantic nodes in our work to construct a variety of different bipartite graphs.
Cui et al., 2020, [14]	Topic-GraphSum	It uses a BERT model that creates a graph-based model of sentence coding and obtaining information on a hidden subject. This topic information acts as an additional semantic unit using a combined neural network (NTM) model.
Huang et al., 2021, [15]	DiscoCorrelation-GraphSum	Different graph formats were proposed and used three types of nodes: sentence locations, EDU locations, and business locations, and RST speech separation to capture interactions between EDUs and to use external speech information to improve model outcomes.
Proposed	N-GPETS	Our attention to a neural heterogeneous graph-based statistical model of pretrained pretraining builds strong relationships between sentences based on additional semantic keywords (sentence-word-sentence). Due to the classification of nodes, sentences are specifically selected to produce our proposed N-GPETS model.

**Table 5:** ROUGE *F*1 scores/results on the CNN/DM data set.

Models	CNN/Daily Mail		
	R-1	R-2	R-L
Lead-3	40.42	17.62	36.67
Oracle	55.61	32.84	51.88

Non-BERT graph models			
NeuSum	41.59	19.01	37.98
HSG	42.31	19.51	38.74
HSG + tri-blocking	42.95	19.76	39.23
BanditSum	41.50	18.70	37.60
JECS	41.70	18.50	37.90

BERT-based graph models			
BERTSUM (sent)	43.25	20.24	39.63
HiBERT	42.37	19.95	38.83
DISCOBERT	43.77	20.85	40.67
Topic-GraphSum	44.02	20.81	40.55
DiscoCorrelation-GraphSum (EDU)	43.61	20.81	**41.12**
N-GPETS (proposed)	**44.15**	**20.86**	40.97

The bold values against the model shows that the corresponding model gain the highest performance in comparison to all other models listed in table.

**Table 6:** Effect of ablation on different models on CNN/Daily Mail test set.

Model	R-1	R-2	R-L
N-GPETS full (proposed)	44.15	20.86	40.97
-Residual connections	43.41	20.32	40.08
*∗*TF-IDF values	43.22	19.97	40.05
-BERT	42.31	19.51	38.74

The module with the ‘-' was taken out of the original N-GPETS, but the module with the ‘∗' had changes made to it.

## Data Availability

The data that support this study are available upon request from the first author.
